# Assessment of photocatalytic potentiality and determination of ecotoxicity (using plant model for better environmental applicability) of synthesized copper, copper oxide and copper-doped zinc oxide nanoparticles

**DOI:** 10.1371/journal.pone.0182823

**Published:** 2017-08-10

**Authors:** Debadrito Das, Animesh Kumar Datta, Divya Vishambhar Kumbhakar, Bapi Ghosh, Ankita Pramanik, Sudha Gupta, Aninda Mandal

**Affiliations:** 1 Department of Botany, Cytogenetics, Genetics and Plant Breeding Section, Kalyani University, Kalyani, Nadia, West Bengal, India; 2 Department of Botany, Pteridology and Palaeobotany Section, Kalyani University, Kalyani, Nadia, West Bengal, India; 3 Department of Botany, A.B.N. Seal College, Cooch Behar, West Bengal, India; Institute of Materials Science, GERMANY

## Abstract

**NPs synthesis, characterization and azo-dye degradation:**

A facile cost effective wet chemical method of synthesis is proposed for Cu-NPs, CuO-NPs and Cu-doped ZnO-NPs. The nanomaterials are opto-physically characterized for nano standard quality. Cu-doped ZnO-NPs based catalytic system is found to possess most efficient photocatalytic activity in degradation of two organic azo-dyes namely methyl red (MR) and malachite green (MG) that are released as industrial effluents in eco-environment intercollegium. Two possible photocatalytic degradation pathways are proposed to understand the mechanism of interaction prevailing during the mineralization of MR and MG dyes. Such study provides insight for waste water management. The uniqueness of the present work is 1) possible routes of MG dye degradation by Cu-doped ZnO-NPs and subsequent intermediate by-products are novel and pioneered of its kind. 2) two new intermediate byproducts are identified suggesting prevalence of multiple MR degradation pathways by Cu-doped ZnO-NPs.

**Assessment of ecotoxicity:**

For assessment of residual NPs impact on environment, eco-toxicological assay is performed using plant system (*Sesamum indicum* L.) as model. The study encompasses seed germination, seedling morphology, quantification of endogenous H_2_O_2_ and MDA generation, estimation of DNA double strand break and analysis of cell cycle inhibition. Results highlight reduced ecotoxicity of Cu-doped ZnO-NPs compared to the other synthesized nanomaterials thereby suggesting better environmental applicability in waste water purification.

## Introduction

Nanomaterials are significant submicron supra-atomic structures possessing next generation potentiality in multidisciplinary scientific applications [1–2]. Furthermore, nanoscale geometry including high surface to volume ratio, wide exciton binding energy, specialized conductivity, among others empowers metallic, metallic oxide and semi-conductor (QDs) nanoparticles (NPs) with chemo-reactive ability towards the development of green technology dealing with environmental health monitoring and management [3–7]. Among the metal oxide NPs, ZnO-nanostructures exhibit wide morphological diversities like simple ball shape, micro-nano filapodia, tetrapod, needle-topped nanorosette, among others [2,8–9]. Applicational potentiality of such nanoscale structural complexes is significantly assessed based on their photocatalytic [10–14] and UV photodetection and gas sensing [15] ability, antimicrobial [16–19] and anti-cancerous [20–22] potentiality and also for virostatic [23] as well as immune-protective [24] activities among others [25].

Release of organic azo-dyes namely, methyl red (MR) and malachite green (MG) as industrial effluents is a major threat to ecosystem [26]; although, extensively used in paper, rubber, plastic and textile industries [27–28]. About 15.0% of these synthetic azo-dyes are released in waste water during their processing [29–30], and are reported to cause tissue necrosis, heart block and failure, jaundice among others [31]. Different classes of chemical oxidants are conventionally used to eliminate such dye contamination from waste water [32] but high stability of the dyes towards the oxidizing agents [33–34] results in inadequate removal of toxic compounds. Nanomaterials possessing strong chemo-reactive potentiality is used for photocatalytic degradation of organic dyes [35–37], but assessment of reaction mechanism, degradation kinetics and intermediate compound and by-product identification are essential to design a “sense and shoot”[38] based ultimate catalytic system with wide eco-environment implicational feasibility. Moreover, residual nanomaterials released during the process of dye elimination and industrial waste water purification is a potent source of biohazards and can generate ecotoxicity. Toxicological impact and safety assessment of NPs are investigated in mammalian and human cell lines [39–40] but rarely in plant species [41]. The rooted plant species can well be used for assessment of residual toxicity as soil serve as reservoir for released NPs in the eco-environmental inter-collegium. Such toxicological assessment is significant for selection of nanoparticle based catalytic system towards environmental application. Available literatures addressing photocatalytic potentiality of nanomaterials lack the assessment of environmental applicability and needs to be investigated before reaching to a logical conclusion.

Present investigation highlights the objectivity undermined and encompasses wet chemical synthesis (gelatin encapsulated copper, copper oxide and copper doped zinc oxide) and opto-physical characterization (UV-Vis, FTIR, XRD, DLS and FESEM) of novel class nanomaterials. Photocatalytic potentiality of the prepared NPs is primarily assessed under UV-visible-near infra-red spectroscopy. Furthermore, by estimating pseudo first order photocatalytic reaction kinetics and dye elimination half-life, most promising nanomaterial is selected. Based on the identification (using High Performance Liquid Chromatography—HPLC) and quantification (Ultraperformance Liquid Chromatography Electron Spray Ionization Quantitative time of flight-Mass Spectroscopy—UPLC-ESI-QTOF-MS) of intermediate and by-products, a possible reaction pathway is proposed for both the azo-dye degradation. Ecotoxicity of the residual NPs is studied (seed germination, seedling growth and morphology, stress accumulation, genotoxicity and cell cycle inhibition) using plant system (*Sesamum indicum* L., family: Pedaliaceae, common name: sesame; oil yielding plant in commerce) as toxicity analyzing platform.

## Materials and methods

### Preparation of nanoparticles (NPs)

#### Cu-NPs

About 50 ml gelatin solution (5%, w/v) was prepared by adding gelatin powder (Merck) in milli-Q water followed by vigorous stirring for 8 h. Drop-wise addition of 0.01 M copper chloride (Merck, AR) solution in the aqueous gelatin was preceded by inclusion of 0.1 M potassium hydroxide (Merck, AR). Complete reduction of metallic copper was materialized by hydrazine hydrate (0.1 M, 500 μL; Merck, AR) in the reaction system. Resultant suspension was kept undisturbed for 6 h for spontaneous growth of nanoparticles. Nanosuspension was kept in airtight capped container.

#### CuO-NPs

For synthesis of CuO-NPs, copper acetate (0.01 M, Merck, AR), potassium hydroxide (0.01 M, Merck, AR) and 10% (w/v) sodium dodecyl sulphate (SDS; Merck, AR) solutions were prepared separately. Copper oxide nanostructure was grown by dropwise simultaneous addition of copper acetate and potassium hydroxide (1:2) solution in the SDS capping environment followed by microwave exposure (frequency: 2450 MHz; photon energy: 1×10^−5^ eV) for 3 min. NPs preparation was confirmed visually by appearance of blackish brown coloration of the resultant suspension.

#### Cu-doped ZnO-NPs

Copper doping of zinc oxide nanostructures was employed for its photo-reactivation both in visible as well as in UV region of spectrum. For the purpose, zinc acetate (0.01 M, Merck, AR) and copper acetate (0.01 M, Merck, AR) reagents were prepared. Reaction was carried out by adding both the reagents in the micro-wave irradiated potassium hydroxide (0.1 M; Merck, AR) under continuous stirring. Particle growth was visually confirmed by development of milky white coloration of the nanosuspension.

### Characterization

All the prepared nanoparticles were opto-physically characterized for determining their morphology, geometry, crystallinity and electrical property. Instrumentation tools employed were UV-vis near infra-red (Shimadzu UV-1800) and Fourier transform infra-red spectrophotometer (Jasco FT/IR-6300; using IR grade KBr), X-ray diffraction analyzer (Shimadzu LabX), Dynamic light scattering-zeta potential analyzer (Delsa Nano C, Beckman Coulter) and Field emission scanning electron microscope (JEOL JSM 7600-F).

### Measurement of photocatalytic activity

#### Preparation of dye sample

Model dyes namely, methyl red (MR—Merck, AR) and malachite green (MG—Merck, AR) were used to assess the photocatalytic degradation efficiency of the prepared nanosuspensions. For the purpose, methyl red and malachite green solutions (3×10^−5^ M) were prepared using milli-Q water.

#### Experiment

Dye degradation solutions were prepared in microcentrifuge tubes (Tarsons, 2 ml) by mixing dye solution and nanosuspensions (4 μg ml^-1^) in a 9:1 ratio. Resultant solutions were vortexed (Remi CM101 Cyclomixer) and subsequently irradiated under sunlight [solar irradiance (DNI)—5.32 kWh/m^2^/day; source: mnre.gov.in/sec/solar-assmnt.htm] up to 2 h. Reaction conditions of both dye degradation solutions were maintained pH 6.3.

#### Analyses

Photocatalytic degradation kinetics was determined using UV-visible near infra-red spectrophotometer (range: 190 nm to 1200 nm; Shimadzu UV-1800). Identification and quantification of reaction intermediates and end products were performed using High Performance Liquid Chromatography (HPLC; Hitachi, Chromaster with UV-vis detector; flow rate: 10μl min^-1^, solvent: acetonitrile:water::60:40, detection wavelength: 425 nm for MR and 618 nm for MG; C-18 reverse phase column—4.6 mm × 250 mm with 5 μm particle size) and High Resolution Liquid Chromatography Electron Spray Ionization Quantitative time of flight Mass Spectroscopy (LC-ESI-QTOF-MS; Xevo G2-XS QTOF, Waters; C-18 analytical column of 2.0 mm × 150 mm with 3 μm particle size, flow rate: 0.2 ml min^-1^, capillary voltage: 3.8 kV, nebulizer pressure: 50 psi). For HPLC and ESI-MS analyses, reaction suspensions were centrifuged at 12,000 rpm for 15 min.

### Assessment of phytotoxicity

#### Treatment

For phytotoxicity assessment, dry seeds (moisture content: 3.64%) *Sesamum indicum* L. var. B67 (procured from Pulse and Oil seed Research Station, Govt. of West Bengal, Berhampore, India) were soaked in nanosuspensions (1.0, 2.0 and 4.0 μg ml^-1^) for 3 and 6 h durations. NPs treated seeds along with dry control were allowed to germinate in Petri plates lined with moist filter papers.

#### Germination

Germination frequency in treatments was measured on the 7^th^ day from the date of treatment. Radicle emergence was taken as an index of germination.

#### Seedling growth and morphology

Seedling growth (7^th^ day from treatment) along with root to shoot length ratio were measured under Stereo-microscope (Stereo Zoom S8APO, Leica). Morphometric deformities noted in treated seedlings were analyzed and photomicrographed under both Stereo microscope and Scanning Electron Microscope (ZEISS EVO-MA 10).

#### Measurement of stress induction by NPs

Extent of *in vivo* stress generation by nanoparticles was estimated by measuring hydrogen peroxide (H_2_O_2_) [42] and malondialdehyde (MDA) [43] accumulations in NPs treated seedlings.

#### Assessment of DNA double strand breaks by single cell gel electrophoresis

Plant nucleoli isolation and single cell gel electrophoresis were performed according to Pourrut et al [44]. Suitable comet slides were photomicrographed and tail DNA percentage was measured using Comet Assay IV software.

#### Assessment of cell cycle inhibition by NPs treatment

Cell cycle inhibition due to NPs treatment was studied using Flow cytometry. For the purpose, nuclei suspensions were prepared from 7 days old seedlings [45] followed by incubation with 50 μg ml^-1^propidium iodide (simultaneously with RNase—50 μg ml^-1^) and analyzed under Fluorescence assisted cell sorter (BD FACs Verse equipped with band pass filters: excitation: 488 nm; emission: 527 nm; Argon laser). Data analysis was performed using BD FACs Suite^™^ software.

## Results and discussion

### Characterization

UV-visible spectroscopic absorption reveals characteristic plasmon resonance at 585 nm for Cu-NPs (Fig 1a) demonstrating metallic copper as the elemental nature of prepared nanosuspension. Well defined absorption edges at 562 nm and 578 nm are documented for CuO and Cu-doped ZnO-NPs respectively (Fig 1b and 1c). For ZnO-NPs, a prominent notch demonstrating a sharp decline in visible light absorption efficiency at 562 nm is observed and is assumed to be the characteristic signal of copper doping (Fig 1c). Blue shifting of absorption efficiency noted for the prepared semiconductor NPs possibly demonstrate the particle coupling effect [46] as well as quantum confinement [47]. For copper doped ZnO-NPs, absence of sharp red shifting pattern in visible light absorption is possibly the indication of abundant blunt edged ZnO-wurtzite nanocrystal over the typical sharp one [48].

**Fig 1:** Opto-physical attributes of nanoparticles (NPs). (a–c) UV-vis absorption plots showing light absorption efficiency in the visible spectrum region, (d–e) FTIR plot showing transmissional depressions at different wavelength region, (f–h) X-ray diffraction patterns with multiple peak positions at Braggs angles (2θ) demonstrating crystal faces of NPs.

Fourier transform infra-red (FTIR) transmission plot reveals multiple inverse transmission peaks at the region of 426–637 (CuO—stretching), 1539 (C-H vibration), 1628 (O-H deformation), 2880 (O = C = O stretch), 3423 (OH group vibration) cm^-1^ for CuO-NPs (Fig 1d).Cu-doped ZnO-NPs exhibits multiple peak positioned at 563 (Zn-O bond vibration), 1623 (H-O-H bending vibration) and 3459 cm^-1^ (OH group stretching) regions (Fig 1e) demonstrating the chemical bonding nature. Interestingly, localization of weak to medium bands at 638 cm^-1^and 869 cm^-1^ are the possible indication of vibrational frequencies assigned to the altered wurtzite ZnO nanostructure due to Cu penetration in Zn-O crystal lattice.

X-ray diffractogram of the prepared Cu-NPs shows characteristic triplet peaks (Fig 1f) at 43.3°, 50.8° and 72.8° assigned to the respective crystal faces of (1,1,1), (2,0,0) and (2,2,0) demonstrating face centered cubic morphology (FCC) of metallic copper (ICDD 04–0836) [49–50]. Scattering plots of CuO-NPs (Fig 1g) demonstrate [35.6° - (1,1,1)], [38.6° - (1,1,1)] and [53.6° - (2,0,2)] index pattern attributing to spherical to ellipsoidal particle geometry. Distinct peak localization of Cu-doped ZnO-NPs at 2θ values of 32.1°, 34.6°, 36.2°, 47.7°, 59.2°, 63.1°, 66.2° and 68.2° exhibit the existence of (1,0,0), (0,0,2), (1,0,1), (1,0,2), (1,1,0), (2,0,0) and (2,0,1) lattice planes respectively (Fig 1h). Such index pattern demonstrates wurtzite hexagonal type nano morphology of ZnO crystal (ICDD file no. 36–1451).

Particle size distribution curves obtained from DLS analyzer show mean hydrodynamic diameters estimated to be 33.3 nm, 48.2 nm and 79.2 nm for Cu-NPs, CuO-NPs and Cu doped ZnO-NPs respectively (Fig 2a–2c). Zeta potential values are determined as -13.73, -8.37 and -28.23 mV for Cu-, CuO- and Cu-doped ZnO-NPs respectively (Fig 2d–2f). Negative surface charge is the indication of nanoparticle stability in the suspension thereby preventing progressive particle agglomeration [51].

**Fig 2:** Characterization of NPs. Bar histograms documenting particle distribution under DLS (a–e), intensity plots exhibiting surface electric charge potential under Zeta potential analyzer (d–f), FESEM image showing surface morphology and shape of individual nanocrystal (g–i), EDX plot demonstrating elemental nature of nanocrystals (j–l).

Scanning electron micrographs of Cu-NPs (Fig 2g) demonstrates inner metallic core (size: 18.37 nm ± 6.39) along with outer gelatinous shell (64.23 nm ± 22.37) documenting encapsulated copper nanocrystal. For CuO-NPs (Fig 2h), individual submicron (56.47 nm ± 14.20) nanostructures are with spherical to cuboid geometry. SEM observation of Cu-doped ZnO-NPs (Fig 2i) shows typical wurtzite nanorods with partially cylindrical appearance over sharp hexagon thereby indicating the effect of copper doping during ZnO crystal growth [52]. Energy dispersive spectra confirm the basic elemental chemistry of the nanoparticle types (Fig 2j–2l). EDS plot of ZnO-NPs also reveals the presence of copper as dopant within the zinc oxide lattice (Fig 2l).

### Photocatalytic activity

UV-vis near infra-red absorption spectra of MR (Fig 3a, 3c and 3e) and MG (Fig 3b, 3d and 3f) show definite peaks positioned at 425 and 618 nm respectively. In presence of nanoparticles, evolution of spectral band associated with progressive reduction of organic dye is noted under visible light irradiation. Results (Fig 3a–3f inset) demonstrate time dependent catalytic degradation of azo-dyes. Maximum reactivity is observed for Cu-doped ZnO-NPs followed by Cu-NPs and CuO-NPs. Similar result is also observed when catalytic performance of the employed NPs is assessed from the degradation ratio (C/C_0_) of MR and MG over the function of time (Fig 3a–3f inset).

**Fig 3:** UV-visible absorption spectra of MR (a,c,e) and MG (b,d,f) dye degradation reaction mixtures (NPs + azo-dyes) under different time interval upto 60 min. Inset showing NPs mediated time dependent catalytic degradation of azo-dyes (g–h).

Based on Langmuir-Hinshelwood model, inter-relationship is ascertained between the rate of photocatalytic dye degradation and irradiation time. Natural logarithmic plots of the dye ratio (primary concentration and concentration after catalytic degradation [-ln(C/C^0^)]) against corresponding irradiation time yield near linear relationship (Fig 3g and 3h). Such relationship suggests NPs mediated catalytic degradation belongs to pseudo first order reaction kinetics. The first order [53–54] and pseudo first order [30] dye degradation kinetics are also established using different catalytic systems. From the slope of catalytic plots, rate constant is found to be maximum for Cu doped ZnO-NPs demonstrating calculated limiting half-life of degrading dyes (Fig 3g and 3h). Enhanced photocatalytic potentiality of the doped particle relative to pure NPs is attributed towards the production of new energy levels by dopants and increase of life time of electron-hole pairs generation by photon-irradiation [54]. In doped particles, photo-generated electron-holes are trapped by dopant induced defects in the nanocrystal lattice resulting in enhancement of electron-hole pair lifetime and subsequently increase the probability of catalytic reaction between electron-hole pairs and adsorbed dye species [55]

Equations derivatized for the mathematical explanations are summarized below:

i $$-\frac{dC}{dt}=\frac{K_{R}K_{D}}{1+K_{D}C}[K_{D}-adsorption\;coefficient\;of\;NPs,\;K_{R}-reaction\;rate\;constant,\;C-concentration\;at\;any\;time]$$
ii $$ln\left(\frac{C}{C_{0}}\right)=K\;\left(C-C_{0}\right)+K_{R}K_{D}t\;\;\;\;\;\left[\;C_{0}-initial\;dye\;concentration\right]$$
  For pseudo first order reaction, *K*_*D*_*C* is negligible, so
iii $$ln\left(\frac{C}{C_{0}}\right)=K_{R}K_{D}t=Kt\;\;[K=K_{R}K_{D}\text{ is pseudo first order reaction rate constant}]$$
iv $$t_{1/2}=\frac{0.693}{K}[t_{1/2}=half\;life\;of\;organic\;dye]$$

### In vitro ROS generation ability of the NPs

Generation of reactive oxygen species during dye degradation by best performing Cu-doped ZnO-NPs is confirmed by nitroblue tetrazolium (NBT) test as per Bhati et al. [56]. For the purpose, 200 μL NBT along with carbon tetra chloride (CCl_4_) are added to the NPs suspensions. After 1 h of visible light irradiation, reaction mixtures are analyzed under UV-visible spectrophotometer (JASCO V-630) with a functional spectrum of 300 to 800 nm. The absorption plots are presented in Fig 4. NBT test documents color change of CCl_4_ layer from colorless to pinkish violet confirming generation of ROS by NPs and subsequently cause reduction of NBT. Such reduction results in formation of diformazan dye responsible for pinkish coloration.

**Fig 4:** Visible absorption plot documenting degradation of NBT following ROS generation by Cu-doped ZnO-NPs.

### Recycling ability of the Cu-doped ZnO-NS

To evaluate the recycling ability of the best performing Cu-doped ZnO-NPs, the assigned nanocrystals are collected following centrifugation (2000 rpm for 15 min) of dye degradation reaction mixture (after 1 h of solar irradiation). Recovered nanostructures are washed in de-ionized water (for 15 min), sonicated and applied for next round of photodegradation of MR and MG dyes (identical reaction mixtures). The process is repeated upto ten cycles and corresponding dye degradation percentage is measured from UV-visible absorbance data (Fig 5). Considerable photocatalytic efficiency (50% reduction) is noted for upto 6 and 7 cycles of MR and MG dye degradation respectively which clearly indicates the promising reusable potentiality of the Cu-doped ZnO-NS.

**Fig 5:** Per cent of dye degradation by Cu-doped ZnO-NPs after 1 h solar irradiations (using same recovered nanocrystals) after different photocatalytic cycles.

### Mechanism of photocatalytic degradation of organic dyes by Cu doped ZnO-NPs

#### Photon induced activation of NPs

Photocatalytic reaction mechanism of the best performing Cu-doped ZnO-NPs is investigated following the application of HPLC coupled with ESI-TOF-MS and the results obtained are depicted in Figs 6–9. From the mass chromatogram, intermediate compound identification is made from the NIST (National Institute of Standards and Technology, USA) online spectral library (www.nist.gov/pml/atomic-spectra-database).

**Fig 6:** (a-d) HPLC chromatograms showing diminishing tendency of MR dye specific peak at different time interval under Cu-doped ZnO-NPs mediated photocatalysis, (e) UPLC chromatogram consisting intermediated by-product peaks at 30 min irradiation exposure. (f–i) ESI-MS plots of UPLC fractions showing abundant compounds at the specific elution time.

**Fig 7:** Proposed MR degradation routes by Cu-doped ZnO-NPs.

**Fig 8:** Photocatalytic degradation mechanism of MG by Cu-doped ZnO-NPs. UPLC chromatograms of dye degradation reaction mixture at 0 min (a) and 30 min (b) of solar irradiations, (c–e) ESI-MS spectra of UPLC peak fractions (showing relatively abundant by-products compound).

**Fig 9:** Proposed routes of MG mineralization by Cu-doped ZnO-NPs.

Mechanism of photocatalytic degradation of organic dyes by Cu doped ZnO-NPs is attributed towards the photo activation of the nanocrystal surface. By the flash of visible light (containing 5–10% UV irradiation), photons strike the surface of ZnO resulting in excitation drive of electrons from its valance band to conduction band leading to formation of photo generated electron hole. Excited electrons in conduction band produce photocatalytically active reaction centres over the surface of wurtzite nanocrystals. Presence of copper dopant on the nanostructure surface increases the free electron affinity of the reaction system.

$$ZnO\;+\;h\upsilon \;\to \;ZnO^{ex}\;-\;h_{v}^{+}$$

Valance band containing photo generated holes readily reacts with system water forming protonated hydroxyl [OH**˙**] radicles which in turn lead to chemo-degradation of organic dyes.

$$H_{2}O\;⇌\;H^{+}\;+\;OH^{-e}$$

$$OH^{-e}\;+\;h_{v}^{+}\;\to \;OH˙\;+\;ZnO\;-\;h_{v}^{st}$$

OH˙ + Dye → Dye degradation

In a simultaneous 2^nd^ reaction pathway, valence band hole along with charged conduction band-orbital unbiasedly react with electron donor (dissolve oxygen) and electron acceptor (oxygen radicles) respectively which subsequently generate unstable super anionic radicles including superoxides ($O_{2}^{-}$) as well as $HO_{2}^{.}$. These super active radicles serve as possible reaction vessels for mineralization of complex dye compounds.

$$O_{2}\;+\;ZnO^{-e}\;\to \;O_{2}^{-.}$$

$$O_{2}^{-}+\;H_{2}O\;\to \;HO_{2}^{.}+\;OH^{-}$$

$$HO_{2}^{.}+\;ZnO^{ex}-h_{v}^{+}\;\to \;OH^{.}$$

$$OH^{.}\;+\;Dye\;\to \;Low\;molecular\;weight\;compounds$$

Presence of copper ion (due to its high electron affinity) on the wurtzite nanocrystal surface possibly supports the generation of OH**˙** radicles resulting in enhance photocatalytic performance of the nanoparticles. At the time of catalytic activity, ionic coppers are adsorbed on the NPs surface forming the metallic copper from its cationic precursor. Therefore ionic copper act as barrier against recombination of opposite charges localized in conducting and valance band of the nanocrystal and favors the generation of OH**˙** radicles in the reaction system [30]. Retardation of such electron-hole recombination by surface deposited copper particles increases the catalytic efficiency of ZnO-NPs. The said reaction kinetics is favored thermodynamically due to the higher fermi level of ZnO than Cu [57]. Similar findings are also reported comprising different class of semiconductor (CdS, SnO, TiO_2_, ZnO among others) particles [30,58–59]. However possible effect of copper doping on photo-reactivation of blunt edged hexagonal ZnO nanocylinder is reported for the first time.

#### Dye degradation by activated NPs

**Methyl red (MR)**: Hydroxyl radicles (OH**˙**) produced on the nano platform possibly act as primary reactant with MR. Resultant dye by-products are identified by HPLC-QTOF-MS analyses of the reaction mixture. According to the HPLC chromatogram coupled with mass spectrum, two separate degradation route (Fig 7) is possibly in operation parallely. First route involves in OH**˙** mediated homolytic break-down of carbon-nitrogen bond of amine group resulting in formation of methyl group substituted intermediate 1^MR^ (dehydrogenated product). Reaction is further progressed by substitution of second methyl group with hydrogen atom resulting in formation of photolytic by-product (intermediate 2^MR^). Second degradation route is prevailing by opening of aromatic benzene ring by hydroxylation. Existence of intermediate compounds consisting hydroxyl substituted dimethyl amino group containing benzene ring supports the catalytic pathway. Such hydroxylated products are responsible for peak broadening in MR spectrum [60]. Low molecular weight [m/z 92, 97, 108, 120, 139, 148, 197] by-products formed during catalytic degradation of MR dye contributes to blue shifting of absorption spectrum compared to non-degraded MR dye. Further reaction progresses upto 60 minutes in a recurrent fashion before complete mineralization of aromatic dye.

**Malachite green (MG)**: Cu doped ZnO-NPs mediated MG degradation involves two simultaneously occurring photolytic routes (Fig 9). First recurrent OH**˙** attack reaction involves in the serial substitution of methyl group by hydrogen atom resulting in the formation of reaction intermediates (m/z 315, 301, 287, 273). In the second reaction pathway, hydroxylation coupled with demethylation results in production of (methyl amino phenyl)-phenyl methanon [m/z 212] which is further degraded towards the formation of (amino phenyl)-phenyl methanon [m/z 197] by methyl group substitution reaction. Further photocatalysis involving aromatic ring opening by hydroxyl group is operational [m/z 107, 132, 136, 181] before complete mineralization and decoloration of MG. The proposed mineralization pathways of MG dye by Cu-doped ZnO-NPs comprising intermediate by-products are novel and reported for the first time in literature.

### Assessment of phytotoxicity

#### Germination frequency

Germination frequency is found to reduce in NPs treatments (Cu-NPs: 70.0% to 48.0%; CuO-NPs: 72.0% to 52.0%; Cu-doped ZnO-NPs: 72.0% to 58.0%) than control (80.0%) and the reduction is mostly dose dependent. Reduction is is in the following order: Cu-NPs>CuO-NPs>Cu-doped ZnO-NPS. However, none of the employed doses of NPs show 50.0% inhibition in germination.

#### Seedling growth and morphology

Excepting Cu-doped ZnO-NPs, significant (p<0.05, evinced from CD determination) inhibition (Fig 10a) in seedling growth is noted in NPs treatment compared to control. Similarly, reduction in root-shoot ratio is observed in treatments (Fig 10b). Data across doses of NPs demonstrate that seedling length suppression is in the following order of CuO-NPs≈Cu-NPs>Cu-doped ZnO-NPs.

**Fig 10:** Assessment of phytotoxicity induced by NPs. Seedling length (a) and root to shoot index (b) in different NPs treated seedlings compared to control. Stereomicroscopic images showing morphological deformities in seedlings induced by NPs (f–k) compared to controls (c–e).

Bright field Stereo-zoom (Fig 10c–10e–normal; Fig 10f–10k–treated) and scanning electron micrographs (Fig 11a–11f) of treated seedlings in relation to controls (Fig 10c–10e) reveal different morphological anomalies. The abnormalities studied are radicle bifurcation (Fig 11b), root cap deformation (Fig 10i–10k), root hair suppression (Fig 11a), radical necrosis (Fig 10f–10g), plumule browning and necrosis (Fig 10h), shrinking (Fig 11c), leaf epidermal rupturing (Fig 11e and 11f) and leaf surface lesion (Fig 11d). NPs mediated reduction of root:shoot index is possibly the indication of stunted radical growth leading to seedling length suppression and desiccation.

**Fig 11:** Scanning electron micrographs showing structural anomalies in seedlings induced by nanoparticles.

#### Measurement of stress

Quantification of H_2_O_2_ and MDA in treated seedlings (data pooled across doses of treatment) reveals higher stress responsiveness of CuO-NPs (Fig 12b) than Cu-NPs (Fig 12a). Cu-doped ZnO-NPs is unable to demonstrate any significant contribution towards stress generation in relation to control (Fig 12c). Relatively larger particle size of ZnO-NPs may be the contributing factor for lesser reactivity with the biological interface.

**Fig 12:** Comparative assessment of stress induction (in the form of H_2_O_2_ generation and MDA formation) in seedlings by nanoparticles.

#### Assessment of genotoxicity by single cell gel electrophoresis

Data exhibits mostly dose dependent enhancement in percentage of tail DNA suggesting double strand break mediated by NPs (Fig 13a). Estimated tail-DNA per cent in different doses of NPs (Fig 13c–13g) in relation to control (Fig 13b) suggest genotoxicity. DNA damaging potentiality across doses of NPs is found to occur in the order of CuO>Cu-NPs>Cu-doped ZnO-NPs. Regression analyses also highlight minimum genotoxicity of Cu doped ZnO-NPs (Fig 13a).

**Fig 13:** Comet photomicrographs (% tail DNA) in (a) control and in (b-f) NPs treatments.

#### Flow cytometry

Flow cytometric observation demonstrates that in relation to control (Fig 14a), three distinct NPs mediated negative influence on normalised cell cycle dynamics (Fig 14b–14e) are observed. They are cellular metabolic peak shifting, G_1_ phase blocking and apoptosis. At the initial doses of NPs treatments, metabolic peak shifted towards S/G_2_ segment of cell cycle. Such type of cell cycle distribution is the possible indication of cellular metabolic attempt to overcome NPs generated toxicity on the phytological system. However, higher dose of NPs (excepting Cu-doped ZnO-NPs) results in arrest of cell cycle at G_1_ phase producing blockage on cell cycle progression and subsequent growth and morphogenesis. Varied degree of apoptotic event is also documented in terminal (4.0 μg ml^-1^, 3 and 6 h) and sub-terminal (2.0 μg ml^-1^, 3 and 6 h) doses of treatments (excepting Cu-doped ZnO-NPs). Cu-doped ZnO-NPs show minimum percentage of apoptotic cell death in comparison to other employed NPs (Fig 14f).

**Fig 14:** Assessment of cell cycle distribution pattern of root tip nuclei in control (a) and in NPs treatments (b-Cu-NPs; c,d-CuO-/NPs; e-ZnO-NPs) following flow cytometric analysis. (f) Bar histogram representing percentage of tail DNA formation in NPs treated root tip cells.

Therefore, NPs mediated stress and toxicity is found to be responsible for significant deviation of conserved cellular events.

## Conclusions

The present work is summarized in Fig 15. Cu-doped ZnO-NPs is found to possess most efficient photocatalytic activity compared to Cu- and CuO-NPs. Two possible photolytic degradation pathways are proposed to understand the mechanism of interaction prevailing during mineralization of MR and MG dyes. The novelty of the present work lies in 1) identification of two new intermediate by-products during catalytic break down of MR dye suggesting possible prevalence of multiple interconnecting routes for dye degradation;2) MG degradation routes prevailing during Cu-doped ZnO-NPs induced photocatalysis is pioneered of its kind and 3) assessment of residual NPs impact on eco-environmental intercollegium using plant system (*S*. *indicum*) as model(seed germination, seedling morphology, quantification of endogenous H_2_O_2_ and MDA generation, estimation of DNA double strand break and analysis of cell cycle inhibition) highlightsminimumecotoxicity of Cu-doped ZnO-NPs compared to the other synthesized nanomaterials.Results suggest better environmental applicability of Cu-doped ZnO-NPs in waste water purification. Furthermore, the prepared nanomaterials (Cu-, CuO- and Cu-doped ZnO-NPs) are cost effective, devoid of any complex instrumentation for synthesis and are of international nanostandard quality.

**Fig 15:** Overview of the present investigation.
